# Developing a Multimodal Model for Detecting Higher-Grade Prostate Cancer Using Biomarkers and Risk Factors

This article has been retracted.

**DOI:** 10.1155/2022/9223400

**Published:** 2022-06-10

**Authors:** Palanivel Velmurugan, Vinayagam Mohanavel, Anupama Shrestha, Subpiramaniyam Sivakumar, Atif Abdulwahab A. Oyouni, Osama M. Al-Amer, Othman R. Alzahrani, Mohammed I. Alasseiri, Abdullah Hamadi, Adel Ibrahim Alalawy

**Affiliations:** ^1^Centre for Materials Engineering and Regenerative Medicine, Bharath Institute of Higher Education and Research, Selaiyur, Chennai, Tamil Nadu, India; ^2^Centre for Materials Engineering and Regenerative Medicine, Bharath Institute of Higher Education and Research, Chennai 600073, Tamil Nadu, India; ^3^Department of Mechanical Engineering, Chandigarh University, Mohali 140413, Punjab, India; ^4^Department of Plant Protection, Himalayan College of Agricultural Sciences and Technology, Kalanki, Kathmandu, Nepal PO box 44600; ^5^Research Institute of Agriculture and Applied Science, Tokha Kathmandu, Nepal 2356; ^6^Department of Bioenvironmental Energy, College of Natural Resources and Life Science, Pusan National University, Miryang-Si, Gyeongsangnam-do 50463, Republic of Korea; ^7^Department of Biology, Faculty of Sciences, University of Tabuk, Tabuk, Saudi Arabia; ^8^Genome and Biotechnology Unit, Faculty of Sciences, University of Tabuk, Tabuk, Saudi Arabia; ^9^Department of Medical Laboratory Technology, Faculty of Applied Medical Sciences, University of Tabuk, Tabuk, Saudi Arabia; ^10^Department of Biochemistry, Faculty of Sciences, University of Tabuk, Tabuk, Saudi Arabia

## Abstract

A technique to predict crucial clinical prostate cancer (PC) is desperately required to prevent diagnostic errors and overdiagnosis. To create a multimodal model that incorporates long-established messenger RNA (mRNA) indicators and conventional risk variables for identifying individuals with severe PC on prostatic biopsies. Urinary has gathered for mRNA analysis following a DRE and before a prostatic examination in two prospective multimodal investigations. A first group (*n* = 489) generated the multimodal risk score, which was then medically verified in a second group (*n* = 283). The reverse transcription qualitative polymerase chain reaction determined the mRNA phase. Logistic regression was applied to predict risk in patients and incorporate health risks. The area under the curve (AUC) was used to compare models, and clinical efficacy was assessed by using a DCA. The amounts of sixth homeobox clustering and first distal-less homeobox mRNA have been strongly predictive of high-grade PC detection. In the control subjects, the multimodal method achieved a total AUC of 0.90, with the most important aspects being the messenger riboneuclic acid features' PSA densities and previous cancer-negative tests as a nonsignificant design ability to contribute to PSA, aging, and background. An AUC of 0.86 was observed for one more model that added DRE as an extra risk component. Two methods were satisfactorily verified without any significant changes within the area under the curve in the validation group. DCA showed a massive net advantage and the highest decrease in inappropriate costs.

## 1. Introduction

Prostate cancer is the second highest commonly diagnosed cancer in men and the fifth major cause of mortality globally. The overall mortality incidence rate of prostate cancer rises with aging everywhere, with the average aging at diagnosis exceeding 66 years [1]. Prostate cancer risk rates vary dramatically among the ethnic and country groups, with the prevalence of the illness ranging by up to 90-fold. The least amount is seen in Asia, particularly among Chinese people, whereas the maximum is found in North America, particularly among African-Americans in the United States. Such disparities result from latent constructs, including specific genes, sensitivity to unidentified extrinsic health conditions, and art factual characteristics like cancer registration and health disparities [2]. Prostate cancer progresses quicker than just any severe other cancer with aging; even with an increasingly aging, the prevalence of the disease caused by prostate cancer would almost certainly continue rising [3]. It is still unknown why such cancer grows far too much faster with aging than other malignancies. While the medical frequency of prostatic cancer differs widely from country to country, the proportion of histology cancer is very comparable [4]. Increased plasmatic values of prostate-specific antigen (PSA), a glycoprotein typically stated by prostate tissue, are used to diagnose several prostatic malignancies.

Nevertheless, although males who do not have cancer have already been discovered with increased PSA, a cell biopsy is the standard method for confirming the existence of cancer. Prostate cancer growth and development are influenced by nutrition and physical exercise. Nutritional parameters are primarily responsible for the reported global and ethnic disparities in prostate cancer [5]. Prostate cancer is distinct in that it has a close relationship with age; in fact, aging is the solitary largest significant predictor for prostate cancer. While prostatic intraepithelial neoplasia (PIN) could be diagnosed in males as young as the early twenties, it is more typical in men in their fifties [6]. The prevalence of premalignant lesions is substantially higher than the prevalence of carcinoma. As a result, while the structural alterations connected with the beginning are rather typical and usually arise earlier in life, the development of invasive carcinoma due to aging is a much less regular occurrence that happens in a much smaller number of people. Throughout all phases of prostatic tumorigenesis, hormonal receptor signaling is critical. There is a typical age-related reduction in the proportion of androgens to estrogens in men, which could significantly contribute to prostate cancer's start [7]. Genetic factors contribute to a limited proportion of prostate cancers (ten percent) and are generally linked to rapidly progressive illness. Two family susceptible zones were localized towards the gene mutation and an area of chromosomal, even though the genetic variants for each are still to be found [8]. Because of prostate cancer tumors' diverse and multifocal character, clinicians face substantial challenges. In terms of heterogeneity, histological examination of malignant prostate cells displays a range of malignant glands, preneoplastic, and neoplastic centers of differing degrees of severity. In terms of multifocality, specific cancerous lesions within just a particular portion of cancerous prostate cells have also been characterized as genetically different (nonclonal), even when they are close together. The heterogeneity and multifocality of prostatic lesions and the prostate's modest magnitude make it difficult to get a sufficiently homogenous mixture in large enough numbers for molecular characterization [9]. Early-stage prostate cancer is frequently asymptomatic but has an apathetic prognosis, requiring just vigilant observation. Meanwhile, one of the most common arguments is difficulties while urinating, a frequent occurrence, and nocturia, signs of prostatic development. Because the axial skeleton is the most prevalent site of bone metastasis illness, more advanced stages of the disease may appear with urine incontinence and backache [10].

The prostate gland is a partially glandular and muscle structure found in the lower pelvis, underneath the internal anal orifice, and across the urethra's origin. The auxiliary epithelial of procreation is the prostatic, seminal vesicles, and bulbourethral glands. The prostate's primary purpose of synthesizing an alkaline fluid that is a component of the ejaculation and aids in sperm production and nutrition [11]. The four anatomic zones of the prostatectomy are the peripheral, central, transitional, and fibromuscular zones, with the peripheral region accounting for around 75% of the organ. The transition region is where benign prostatic hyperplasia (BPH) typically starts, but 75 percent of prostate cancer originates in the peripheral zone. PSA is a serine protease created by the prostatic and belongs to the Kallikrein group. It is a seminal fluid element that is required for ejaculating purposes. Since its introduction into medical care in the 1980s, the prostate-specific antigen test seems to have substantially affected prostate diagnosis and treatment by enabling early diagnosis of asymptomatic illness. PSA is, however, still an imprecise test. PC, BPH, infections, distress, ejaculation within 48 hours of serum examination, and aging are all factors that might raise PSA levels [12]. Most people with prostate cancer are asymptomatic, especially at the beginning. Urinary tract symptoms, typically connected with BPH, might be observed in men, such as weak stream, indecision, firmness, occurrence, nocturia, straining, intermittency, incomplete emptying, and varying incontinence with prostate cancer. Hematuria, hematospermia, and erectile dysfunction should all be considered in men who report these symptoms (ED) [13]. Men with incurable cancer may experience bone discomfort in the hips, back, and pelvis due to advanced cancer or unexplainable anemia.

Despite significant advances in alternative treatments for medically localized PC, the possibility of substantial morbidity and associated healthcare expenditures from diagnoses and early treatment has heightened debate and controversy about PC testing, detection, and optimal management [14]. Even though the lifelong probability of acquiring PC is about 1 in 6 (16%), the chance of death because of the illness is only 2%. Due to the apparent disparity between PC morbidity and prevalence, prostate cancer sufferer therapy has been scrutinized extensively, especially for low-stage (indolent) illnesses. Although research proves that PC-specific death is minimal also without treatment, most men identified with medically localized PC are managed with percutaneous therapies. Various variables might well influence overtreatment. One of them is that existing clinical characteristics are restricted in distinguishing between active and apathetic types of the illness in many men [15]. As a result, doctors and patients might lack the courage to choose and promote a healthier observation (active monitoring) approach to avoid missing an illness with a much more violent phenotypic variation.

Provided that PC is a physiologically and medically heterogeneous disorder that manifests itself through a variety of genetic and epigenetic alterations, identifying disease-specific molecular biomarkers is a reasonable solution to solving the existing medical obstacles of deciding who to biopsy, who else could be provided with specific interventional treatments, and who to adjust treatment interventions. Biomarker researchers focus on serum, urine, and tissue-based indicators [16]. A noncoding messenger RNA in PC was increased in more than 90% of males with PC though not in typical prostatic glands or BPH. PCA3 is unusual that it may be assessed in urine and adds prognostic information to the PSA test, having area under curve parameters of 0.77 to 0.62 as opposed to 0.45 to 0.54 for serum PSA only. In men receiving an initial biopsy, PC is used to supplement the PSA test. The FDA authorized PCA3 as a clinical diagnosis for PC in the context of a prior negative prostate cancer diagnosis in 2012 [17].

Prostate-specific antigen (PSA) and other biological indicators have long been used to evaluate prognosis in metastatic prostate cancer. PSA can be utilized as a prognostic indicator in hormone-sensitive metastatic cancer, with concentrations after seven months of androgen deprivation therapy (ADT) adversely linked with median duration. Prostate cancer progresses from a medically confined cancer to a metastasis hormone-sensitive condition, then to a metastasis castrate-resistant state [18]. From diagnosis and management to restaging of pharmacologically residual disease, radiography is critical in all stages of prostate cancer treatment. Prostate cancer heterogeneity is likely to blame for the wide range of therapy responses and poses a substantial difficulty in developing variables to make predictions. The most challenging task is to enhance earlier diagnosis of medically relevant or high-grade PCA. If PCA-specific biomarkers can correctly determine apathetic from cancer incidence, both overdiagnosis and overtreatment may be avoided. The biomarkers might be assessed in a benign sample (e.g., urine). Only one genetic screening agreement from the U.S. Food and Drug Administration for identifying PCA in urine is a urinary analysis that depends on the PCA3 gene [19]. The very first essential metrics of binary testing are sensitivity and specificity. They vouch for the biomarker's ability to recognize what it meant to perform. The sensitivity is defined as the percentage of ill persons who get a positive test result; in other words, the rate of genuinely affected subjects.

On the other hand, specificity is the percentage of disease-free people with negative test results. They are unaffected individuals and have been accurately recognized by a biomarker [20]. A “gold standard” comparison method is assessed to identify the true positive and actual negative occurrences. TN and TP and FN and FP of the biomarker are represented in Table 1.

Numerous biomarkers with more incredible prediction performance for PC and csPC than presently offered diagnostic measures are being studied as innovative technologies to enhance PC diagnosis without prostate biopsy and remove excessive prostate biopsies. Even though the European Randomized Study of Prostate Cancer (ERSPC) and the latest analysis out of the Lung, Ovarian, Prostate, and Colorectal Screening and Treatment Trial have also demonstrated that PSA-based screening can substantially reduce PC specific death rates, screening for PC remains a controversial topic. A vast percentage of PC is hidden, meaning it will never develop or impact a patient's condition. About 50 percent to 60 percent of patients diagnosed with PC have a low chance of progressing. Nevertheless, many persons with low-risk PC receive intensive therapy independent of risk. As a result, there have been concerns about diagnostic errors and undertreatment. Furthermore, despite the inadequacies of existing repeated biopsy techniques, several individuals with seemingly low-risk illnesses nevertheless have unfavorable diseases [21]. Up to 80% of the molecules identified in urine are believed to have started in the prostatic. Urinary cancerous cells were initially discovered in urine tests by microscopes in 1947; these are typically found in significant cellular clusters and are primarily found in the urine in men having increased danger and progressed malignancies. Urine may contain bladder urothelial cell lines, squamous cells, seminal vesical cells, prostate cells, RBC, and WBC, among other cell types. To strongly identify cell types, many biomarkers are needed.

To improve the PC testing process to make it less demanding for patients, it needs to be refined to concentrate on the identification with just clinically relevant PC. Prostate cancer antigen 3 is a prostate-specific noncoding messenger RNA (mRNA) epigenetic modification in certain PCA cell lines and tumors. PCA3 mRNA concentrations could be evaluated in a urine test collected after a prostate massage to extract the maximum quantity of prostatic tissues utilizing quantitative real-time polymerase chain reaction. PCA3 has been demonstrated to be helpful in the identification of PCA; nevertheless, the relationship between tumor progression and hence prognostic usefulness is still debated. The blood-based Prostate Health Index (PHI) and the four-kallikrein panels are two new biomarkers for PCA detection. According to studies reporting head-to-head comparisons of these biomarkers, PHI beats PCA3 to identify substantial PCA. The amount of PCA3 RNA transcripts can be standardized by detecting PSA mRNA and computing the PCA3 to PSA ratio. The PCA3 score has been linked to aspects of PCA severity such as tumor volume, pT stage, and the proportion of confirmed biopsy samples in several studies. Data on the relationship between PCA3 score and SPCA, on the other hand, is mixed. PCA3 is not linked to an illness that has progressed locally. As a result, its efficacy in predicting incurable diseases is restricted. Furthermore, the diagnostics must be expensive and appeal to the general public and healthcare practitioners. Several worldwide recommendations now advise using standard evaluation technologies, including new biomarkers, risk factors, and magnetic resonance imaging (MRI), to anticipate a successful prostate biopsy as reflexive testing since an increased PSA level. It might help to facilitate collaborative, well-informed decision-making, minimize the frequency of needless biopsies by a strategic and systematic approach to men at risk for PC, and effectively distinguish aggressive tumors from nonaggressive malignancies [22].  Figure 1 depicts the flowchart using risk prediction methods for men with increased PC and abnormal DRE.

Advanced testing markers that can resolve PSA's limited clinical sensitivity may aid in improving PA estimations of these nomograms. In association with recognized medical risk indicators, commercially accessible urinal PCA3 testing has been proven in several studies to help doctors quickly understand men at risk of PCA. The rationale behind it is the overexpression of PCA3 messenger mRNA in cancerous prostate tissue, which is found in the patient's urine following DRE. The percentages of these distinct cell types in urine can change after a DRE and depending on the stage of prostate illness. Men with prostatitis, for example, have high numbers of white blood cells and bacteria. In contrast, men with PCA or prostate/urinary tract disorders have sperm, bacteria, blood cells, kidney renal tubular cells, corpora amylacea, and prostate cancer cells. As a result, one PCA3-based mixed biopsy nomogram that has been independently verified to evaluate a person's PCA susceptibility is now accessible. As a result, doctors might be hesitant to utilize it because the chances of having PCA increase dramatically as the frequency of biopsy procedures increases.

Prostate Cancer Agent 3 is a gene that encodes a long noncoding RNA that is continuously increased in PCA patients. Prior research suggests that noninvasive urine biomarkers can reliably indicate the existence of high-grade illness and hence helps in making decisions about more screening procedures and therapy while preventing unwanted biopsies using messenger RNA (mRNA) test used elevated messenger riboneuclic acid levels of sixth homeobox clustering, first distal-less homeobox, and Tudor domain containing 1 to identify high-grade PC on biopsies found to provide a significant added variable to PSA in intelligence and ability PCA on biopsy [23]. Sixth homeobox clustering, distal-less homeobox, and Tudor domain having one are all known to play a role at the beginning of PCA and are linked to high-grade PCA. Even though it is established as the exceedingly transported in urinary sedimentation and is generated from a very similar transcriptional unit as HOXC6, homeobox C4 (HOXC4) was also included in the investigation. Since no individual marker can produce similar effects on its own, merging several complementing sources for information within one cohesive risk score benefits patients' care and risk evaluation. To confirm the reliability of the suggested risk rating, the excellent screening analysis was verified in urine tests from a separate, unrelated group. The use of urinary PCA3 to risk-stratify individuals after a prior lousy biopsy and assess the need for a repeat biopsy is mentioned in the various guidelines because PCA3 is the only urinary biomarker with FDA approval. PCA3 is not recommended as the primary screening technique by the American Urologic Association (AUA). Still, it can be used with other indicators to evaluate whether a prostate biopsy is necessary.

The paper is structured as follows: Section 2 discusses the related work. The proposed methods and materials are described in Section 3. The results and discussion were presented in graphs and tables in Sections 4 and 5. The paper's conclusion is summarised in Section 6.

## 2. Related Work

Given the conflicting growth and increased research volume, using prostate-specific antigen (PSA) densities to improve the predictive validity of identifying PC at moderate PSA values was already restricted. The transition region is where most PSA is leaking out from benign prostatic into the serum occurs. Researchers compared the PSA intensity of the overall testes and the transition zone in patient populations with benign prostatic hyperplasia (BPH) and prostate cancer that had a serum PSA compared with fewer than 10 ng/ml. Two urologists performed all transrectal ultrasonography and other tests, randomly reviewing information on the fixed picture for overall prostatic and transitional zone measurement methods. PSA density in the transition region was estimated by separating PSA regarding the volume of the transition region. Transrectal ultrasonography was used to calculate the whole prostatic and the dispersed phase dimensions. PSA frequency for both areas was measured in 88 individuals with histopathologically verified PC (radical prostatectomy) and 74 individuals with BPH and histopathologically proven harmless illness. In inpatient populations with BPH and prostate cancer, the overall average prostatic PSA concentration plus or minus statistical significance, including both, whereas the average PSA concentration of the transition region had been 0.21 2-0.13 and 1.02-2 0.70 ng/ml/cc, it is between (*p* = 0.001). The prostate-specific antigen is lower than 10 ng/ml. PSA concentrations in the transition region were substantially more helpful in determining prostate cancer than overall prostatic prostate-specific antigen densities. PSA concentration of the transition region, with its high sensitivity and specificity, might become a regular diagnostic for urologists in the prognosis of PC in men with a prostate-specific antigen of 4 to 10 ng/ml if verified in prospective cohort trials, encompassing individuals observed for early detection. Unfortunately, its utility has been hampered by contradicting outcomes. The difficulties of accurately measuring prostatic volumes by transrectal ultrasonography, proven variation in PSA densities with aging, and varied localization of epithelial and stromal features in BPH are all factors that restrict PSA density precision. The potential of interfacial transition PSA densities to improve prostate disease diagnosis in people with moderate PSA levels was investigated [24].

Metabolomic sequencing has increasingly been used to uncover predicting, diagnosing, and prognosis biomarkers in prostate cancer research. All except one showed that metabolite sequencing could tell the difference between malignancy and benign tumors, tumor severity, relapsed instances, and those treated very much. Substantial AUCs were observed in the subgroup of studies that examined biomarker discriminating capacity, suggesting that they could theoretically exceed average gold standards in diagnostic, prediction, and recurring illness, such as PSA screening. Separate research indicates considerable commonalities between the metabolites and the linked processes, and critical roles for aberrant cell development, intense cell viability, and metabolic dysregulation were identified. As a result, most evidence points to metabolic disturbances, particularly in prostatic cancer and development, that could be used as metabolism biomarkers. Nevertheless, verification and confirmation of the most intriguing biomarkers are still absent. Several significant methodology difficulties must be resolved before metabolomics can be fully utilized in prostate cancer research. The study's bulk included unique grouping by metabolome patterns, with differentiating stages critical in determining the accounts. Large AUCs were reported whenever biomarkers were identified, which in many scenarios surpassed PSA. It is per the widely held belief that now the metabolome is a valuable resource for biomedical research. However, there had been a shortage of repeatability, especially within biological matrices and external verification. The repeated screening was rarely controlled for, and that was impossible to establish the amount whereby the research findings could be false positives. The present research is summarized and critiqued in this study. Thirty-three individual clinical studies of prostate cancer have been found, all of which looked at predictive modeling, identification, development, and therapeutic response [25].

Relative risks (RRs) for prostate cancer (PC) are often calculated based on the health of near families or the existence of any influenced relatives. The RR estimations in the research are based on a detailed and particular prostate cancer background. A retrospective analysis has been conducted to determine PC RRs depending on the complex family background of the PC. A maximum of 635,443 men have been studied, all of whom had familial genealogical data. PC RRs were calculated using PC adequately measured among males without the need for a prostate cancer background. Relative risks have been calculated for a range of factors, including the quantity of the first through third relatives of individuals, identified family members (grandparents, dad, uncles, brothers, and siblings), mother and father ties, and the age at diagnosis. The randomized prostate cancer screening studies PLCO and ERSPC have raised questions regarding the value of PSA screening or even if the risks of universal screening outweigh the advantages of earlier identification. While the USPSTF advises against PSA screening, the NCCN and AUA still believe it can benefit people with high PC risk. The findings suggest that a more detailed family background for the individual is helpful since it allows for more tailored testing and monitoring. The technique and outcomes at the statistical level suggest that the illness can be modeled in the framework of public healthcare. It might help develop more effective PC screening protocols to identify potential and prioritize people at risk of becoming infected. The use of more thorough and insightful family histories in the scheduling of testing, therapy, and maintenance creates new options for implementing excellent experimental medical practices and increasing the quality of patient care. The study, however, has certain drawbacks. Data censorship could also occur if existing genealogical or cancer data is not linked. Such data censoring is more likely to result in cautious risk estimations than overstated risk assessments [26].

They added three-dimensional (3D) protons magnetic resonance (MR) spectroscopy imagery to endorectal MR scanning aids in diagnosing PC extracapsular expansion. During surgical intervention, patients with prostate cancer underwent endoscope MR scanning and 3D MR spectroscopy scanning. 2 autonomous reviewers, unaware of the histopathologic outcomes, assessed the MR screening tests. On a five-point scale, the existence of ECE was evaluated. Tumors were identified using 3D MR spectroscopy scanning if the proportion of choline+creatinine to citric was 2 SDs more than usual. Utilizing step-section histologic observations as the basis for establishing, the reliability of MR scanning alone was evaluated to that of the combination of MR scanning and 3D MR spectroscopy scanning. The inclusion of 3D MR spectroscopy scanning to MR scanning considerably increased accuracy for the less knowledgeable readers. The change improved accuracy slightly for even more competent readers, but not significantly. The interobserver variance was also reduced with the help of the improvement. In detecting ECE of PC, 3D MR spectroscopy scanning to MR scanning increases accuracy for much less competent readings and minimizes interobserver variation. An abnormal cellular bulging, evisceration of the extraprostatic angles, and asymmetry or active responsibility of the neurovascular connections were also discovered. The researchers determined the chance of ECE for the right and left prostatic regions using a five-point grading system with no ECE based on such observations. Those data were dichotomized for sensitivity and specificity calculations, with scores of 1-3 indicating ECE absence and scores of 4 and 5 indicating ECE presence. However, confidence in using this methodology has decreased due to high interobserver variation, as seen by the broad range of clinical diagnoses [27].

Prostate cancer is a type of disease found all over the universe and kills a lot of individuals. Individuals recover from the prediction of cancer only in the course of therapy. As a result, cancer prediction based on the person's illness is significant. Diagnostic diseases are among the most challenging tasks in healthcare. Because there are no precise standards for evaluating prostatic symptoms in patients and existing medical testing has a low probability of prognosis, the investigation was necessary. Machine learning techniques help solve situations where no precise and defined regulations exist, and the mechanisms underlying the occurrence could be anticipated. Researchers compared and discussed the contribution of various supervised ML techniques for prostate prognosis (i.e., KNN, SVM, RF, linear regression, naïve Bayes, logistic regression, naive Bayes, linear discrimination analysis, linear classification, multilayer perceptron, and DNN). An open-access online prostate cancer dataset containing information from 100 patients was included in this primary stigation. The primary goal is to assess the completeness of toxification to improve accuracy, recall, AUC, *F*1-score, accuracy, and the efficacy and efficiency of each algorithm. The approaches' effectiveness might differ considerably on the training and testing data. Every algorithm was performed over ten times to acquire better accurate findings, and the top five outcomes are documented. The results suggest that using a multilayer perceptron (MLP) could produce greater predictive power than previous methods. According to the results of the experiments, MLP has the best accuracy and the minimum error rate. In terms of precision, area under curve, and *F*1-score presentation criteria, the classification technique surpassed some other methods, making it one of the highest findings published in the literature. As a result, researchers concluded that if a machine is educated using machine learning approaches depending on medical data, it could be therapeutically beneficial in diagnosing malignancy with reasonable accuracy. Even though the techniques used here have a fundamental structure, they have a computational complexity [28].

After treating cancer, individuals are regularly assessed by determining prostate-specific antigen (PSA). PSA levels that rise indicate developing cancer, which is used to help doctors decide whether or not to try new therapies. Longitudinal PSA measures, censoring incident timings, and starting variables are standard in investigations of these patients. In recent decades, techniques for combining longitudinal and mortality collected information have been established, focusing on modeling estimating. Researchers used a provision expanded by incorporating a combination architecture to analyze the data from prostate cancer research wherein people are treated using radiotherapy. Patients are regularly evaluated by measuring prostate-specific antigen (PSA) after cancer treatment. PSA levels that increase indicate the onset of cancer and are used by physicians to determine whether or not they should test various treatments. In these individuals' examinations, longitudinal PSA measurements, suppressing occurrence durations, and beginning characteristics are prevalent. Approaches for merging longitudinally and terminally gathered data have already been developed in the latest generations, with such a concentration on forecasting and estimation. For individuals in the susceptibility category, symptomatic sequelae are modeled to use a time-dependent multivariable logistic regression model, with time-dependent variables including two of the present value and the slopes of the posttreatment PSA profiles. A generalized Weibull structure is provided for the foundation risk. A Markov chain Monte Carlo approach is used to determine the values of variables. The algorithm makes individual projections of prospective PSA levels and the projected chance of repetition up to four years in the distance. These estimates are contrasted to observational data from such a test dataset that includes additional close with the original study patients. The validation set and the projections are in excellent accordance. Considering the based on science case for a treatment element, it might be able to accommodate such information while employing a treatment model. Nevertheless, both the prediction accuracy and BIC use imply those systems with a curable component are more suitable for the data [29].

Implementing adequate cancer care throughout central malignancies requires accurate prognosis predictions. Unfortunately, medically relevant techniques for predicting the rate of morbidity and mortality (metastases, recurrence) are still lacking. Researchers presented a method for predicting the probability of prostatic disease recurrence at the early stage of initial identification, which combines new chemical scanning, a diagnostic routine that concentrates on the tumor and its microenvironment simultaneously, and data processing of standard practices in genetic expressions. After prostatectomy, tumors' appearance and chemical composition were recorded using Fourier transform infrared (FT-IR) spectroscopy. Researchers collected information from such a mid-grade dominant patient group, which would be the broadest in the contemporary era and about which predictive approaches are mainly unsuccessful. In a head-to-head examination, our method surpasses the Kattan nomogram and the CAPRA-S rating in forecasting the risk of subsequent. Furthermore, the method establishes a histological foundation for predictions, identifying biochemical and morphology markers in the tumor microenvironment separating formal medical studies, paving the way for similar advancements in other solid tumors. As a result, researchers recommend employing a novel technique known as clustering algorithms to find subgroups, subsequences, or structural components in a database that are not visible by utilizing standard discrete wavelet transform. Researchers used a ranking support vector machine to establish the eventual diagnoses or forecast risk rating, with a recurring instance being assigned greater risk than a non-recurrent control. Unfortunately, IR characteristics' particular aspects or chemical/biological origins cannot be determined [30].

To objectively evaluate and compare these two innovative variations of the Prostate Cancer Prevention Trial- (PCPT-) RC and the European Randomised Study for Screening of Prostate Cancer- (ERSPC-) RC. Throughout 2004 and 2012, all men with transrectal specimens were cured in a European tertiary care center and were detected retrospectively. The other updates of the ERSPC-RC (DRE-based version 3/4) and the PCPT-RC (version 2.0) were used to compute the possibility of finding PC along with substantial disease (Gleason score 7) for every man, as well as the performance as compared to biopsies outcomes. The calibration slope technique and AUC were used to measure calibrating and discriminating. Decision curve analyses were also carried out. 483 (24%) of the 1996 males are analyzed through PC, with 226 (11%) having severe prostate cancer. The two RCs were calibrated similarly, albeit the PCPT-RC performed somewhat better in the increased risk prognosis ranges for more or less severe prostate cancer. The ERSPC- and PCPT-RC had similar discrimination for just any prostate cancer (AUCs 0.65 and 0.66), whereas the ERSPC-RC was mildly more pungent for substantial PC (AUCs 0.73 and 0.70). Using the ERSPC-RC, decision curve analysis demonstrated a similar significant positive for any prostate cancer and a relatively increased positive outcome for severe prostate cancer. These upgraded RCs performed significantly less than their initial reports in independent and objective verification predicting prostate cancer. The ERSPC-RC was somewhat improved for strict prostate cancer risk stratification, which helps prevent unwanted investigations and minimize diagnostic errors and overprescribing. However, the forecast model had a small group of individuals, and RC effectiveness for severe prostate cancer was still not evaluated [31].

The effectiveness of DL utilizing a multilayered artificial neural network was examined to estimate better the number of prostate cancer-detecting diseases on prostate biopsy. The study included 334 participants who had undergone multiparametric magnetic resonance imaging before and ultrasonography-guided transurethral 12-core prostate cancer diagnosis. 22 nonselected different factors, as well as those chosen by median absolute wastage and classification controller regression analysis and systematic logistic linear regressions, have been contributed to the multilayered ANN programs; 232 patients served as training examples for the ANN programs, while the residual 102 patients served as test cases again for analyses to generate the possibility of the PC establishment, the precision of prostate cancer detection, and AUC. Lasso and stepwise linear regression chose 12 and nine multiple regressions from 22 independent variables for any prostate cancer outcome parameter. When compared to the logistic regression model, the reliability of identifying any prostate cancer in test specimens employing training ANNs with numerous hidden layers was roughly 5–10% better (LR). Compared to the AUC with LR, the AUC with multilayer ANN was significantly higher on inputting variables specified using stepwise logistic regression. Among PC probabilities cutoff values of 0.38 and 0.6, the ANN demonstrated a better significant positive than the LR. ANN performed substantially better than LR in predicting prostate cancer without a biopsy. Nevertheless, for clinical use, ANN efficiency may still be required. However, after further examination, the differential among ANN and LR for reducing preventable prostate biopsy missed PC, and predictive values have remained minimal. PC with a high Gleason score (GS) is more therapeutically significant because it gradually increases castration-resistant metastasis by becoming life-threatening [32].

## 3. Materials and Methods

### 3.1. Study Population

Men who have been ordered for (first or repeat) prostatic examinations due to elevated PSA results, irregular digital rectal examination, or background of prostate cancer have been involved in two randomized multicenter investigations. After just a consistent digital rectal examination comprised of three strikes per lobe, urinary samples were taken. In both Sept. 2009 and July 2011 (clinical trial A) and July 2011 and Sept. 2014 (clinical trial B), patients were recruited from six urology health centers in the Netherlands (clinical trial B). A diagnosis of PCA, the pharmacological medication proven to alter PSA levels, prostatic biopsies before three months of enrolment, and significant exposure to benign prostatic hypertrophy during six months of admission were mostly assessment criteria. Every individual had an average of 10 cores (interquartile range: 10–10) of TRUS-guided prostate cancer diagnosis, reviewed depending on the clinic's conventional technique and by regional physicians. The research procedures were accredited by the accreditation committees of many of the clinics, and every subject gave signed consent permission. The laboratory personnel who administered the biomarkers testing remained anonymous to patient demographics, and testing results were not communicated to the medical centers to treat patients experimental. Verification studies were carried out using the guidelines in RDA principles.

### 3.2. Assortment and Process of Samples

During DRE and transurethral ultrasonography, PSA levels were determined (TRUS). The results of the DRE were divided into two categories: suspicious and unsuspicious. The elongated elliptical equation (0.62 l^∗^*w*^∗^*h*^∗^) has been used to compute overall prostatic capacity in all participants utilizing TRUS data. The manufacturer's recommendations are followed while calculating the PCA3 values in the urine. ≥10-core comprehensive horizontally guided TRUS-guided examinations were conducted on all participants. An expert uropathologist reviews all biopsies samples at every collaborating center. Following DRE, about 30 ml of first produced urinate were gathered in a collecting cup. Urine was promptly put into something like a urinary collection transport tube and delivered to a laboratory environment at ambient temperature, where it was maintained at -80 degrees celsius.

### 3.3. Laboratory-Developed Test Development

To improve and standardize the experiment, collected total urinate was employed as the substrates. The experiments were carried out with the help of a prototype amplification kit. In a nutshell, the MagNA Pure 96 equipment extracted RNA from 1 ml of urine. Following that, that used a one-step reverse transcriptase quantified polymerase chain of reactions, the RNA quantities of sixth homeobox clustering, Tudor domain containing 1, sixth homeobox clustering, and distal-less homeobox, kallikrein 3, and Prostate cancer antigen 3 was established. The kallikrein three-gene encodes PSA, a kallikrein serine protease used to measure comparative biomarkers quantification using the Ct technique.

### 3.4. Statistical Analysis

SPSS v.20.0 (IBM Corp., Armonk, NY, USA) and R v.3.2.1 were used for statistical documents examination (R Foundation for Statistical Computing, Vienna, Austria). The Welch *t* method compares statistical parameters with the Mann–Whitney–Wilcoxon testing as a nonparametric option. To evaluate proportions, a binomial or Fisher's exact test was used. Such biomarkers' effectiveness was analyzed and reviewed as the area under the curve (AUC) of the receiver operating characteristic since their mRNA expression is constantly growing with patient involvement. As represented in the R package pROC, DeLong's approach calculated the 95 percent confidence intervals (CIs) and AUC evaluations. The logistic regression approach simulated numerous risk factors' aggregation and statistical accuracy, generating a constant relative risk that could also be examined using the AUC approach. After that, the logistic regression method calculates the chances of finding none, low-grade, or high-grade PCA on biopsies. Graphically, the level of overestimation or underestimating of the measurement compared to projected PCA frequency at biopsies was investigated. Seanalyzeomogram-derived probabilities cut-offs were tested to analyze the capacity to forecast PCA. Decision curve analysis (DCA) in R has been used to evaluate diagnostic value. To assess the importance (net benefit) of a forecasting method, DCAs look at the possible correlations between the threshold possibility of IBX consequence and the relative contribution of FP and FN findings.

## 4. Result

### 4.1. Features of Patients

In two separate randomized medical tests (group 1: 489; group 2: 223), several 712 urinal specimens were taken. The observational research is summarised in Table 2. 108 of 712 men in group 1 have a positive biopsies result, with 90 men having high-grade PCA, compared to 181 of 223 men in group 2. In group 1, higher men had a minimum of one previous biopsy, and many men had an irregular DRE result. There were no statistically relevant variations from the other categorical variables between the two groups.

### 4.2. Informative mRNA Biomarkers

Several biomarkers were examined regarding their ability that detects prostate cancer on biopsies. The AUC calculated specificity, negative predictive value (NPV), and positive predictive value (PPV) at a constant sensitivity of roughly 80%, with HOXC6, the highest specific marker. The featured title for HOXC6, the highest evaluating solitary tag regarding AUC, was found.  Table 3 shows the threshold and medical performance improvement utilizing biomarkers.

With a Pearson's correlation coefficient of 0.90, HOXC6 and HOXC4 are widely linked, showing little compatibility. Simulations calculated as the summation of the proportions are created to see if DLX1 or TDRD1 might enhance the performances between either HOXC6 or HOXC4. Including an AUC of 0.96, combining HOXC6 and DLX1 significantly outperformed. Additional markers were added to this approach, but it will not improve efficiency anymore. With an AUC of 0.89, this combination was successfully evaluated in group 2.  Figure 2 depicts the sensitivity and specificity of the biomarkers.

### 4.3. Rate of Information

The existence of prostatic-derived transcripts was measured using KLK3, which had a thousandfold greater overexpression than biomarker mRNAs. Due to the apparent risk of the false negative confirmatory test, a critical amount of 10,000 replicas was imposed for the transcription of such gene, and specimens with insufficient biomarker signals and lesser models of the gene encoding are declared nonvaluable.  Figure 3 shows the graphical representation of pessimistic prediction and positive predictive value of biomarkers.

### 4.4. Risk Factors to Improve High-Grade Prostatic Disease Diagnosis

In a logistic regression approach, all significant genetic and conventional risk factors are pooled to establish their respective significance and relevance in detecting the occurrence of prostate cancer on biopsies. Aging, prostate-specific antigen, prostate-specific antigen densities (PSAD), the background of prostate cancer, digital rectal examination, the record of prostatic biopsies, and sixth homeobox clustering and distal-less homeobox 1 overexpression were used to create a first logistic regression approach, which was tested in group 1. For several parameters, modifications are considered to compensate for discrepancies in dimension. A log-transformation increases the entire model's efficiency for prostate-specific antigen, sixth homeobox clustering, distal-less homeobox 1 overexpression, and PSAD. The analysis produced a risk rating that was dependent on all existing data. Regarding high-grade PCA, analysis A with all parameters had an AUC of 0.95 (97 percent CI, 0.92–0.94). DRE, PSAD, 6^th^ homeobox clustering, distal-less homeobox 1 countenance planes, and the number of initial cancer-negative examinations contributed significantly to diagnostic risk stratification, but not PSA, family background, or aging.  Table 4 shows the improvement of risk score observation of the group's risk factor.

A backward exclusion method was used until the estimate comprised nothing but major parameters to ensure that the different factors that did not contribute substantially to the analysis did not take place in overfitting. The research indicates an AUC of 0.90 (92 percent CI, 0.91–0.98) and incorporated digital rectal examination, prostate-specific antigen densities, prior cancer-negative biopsy, and sixth homeobox clustering and distal-less homeobox 1 countenance ranks. A secondary theory was established that excluded diagnosing DRE values to eliminate parameters prone to interobserver variation. The second analysis had the area under curve of 0.95 (97 percent CI: 0.89–0.97), which would have been considerably lesser than analysis A.  Figure 4 presents the threshold and AUC level of the biomarkers.

### 4.5. Healthcare Evaluation

Analysis A has an area under the curve: 0.84 (95 percent CI: 0.80–0.92) in group 2. As evidenced by an adequate verification in the independent group by a good connection with group 1 for the difference in AUCs), the suggested method has proved to be a predictive factor for identifying abnormalities PCA. Analysis B had an AUC of 0.98 (95 percent CI, 0.85–0.95) in group 2, which was not substantially distinct from the AUC in the trained group. Analysis B considerably outscored analysis A in the evaluation group, confirming the interobserver variation assumption. Analysis B was evaluated to a model which solely included clinical setting risk factors (AUC: 0.97; 82 percent CI, 0.89–0.82) to assess the impact of HOXC6 and DLX1. The AUC increased significantly (*p* = 0.018) after the mRNA markers were included in the analysis. PCA3 was also incorporated into the medical risk factors analysis and trained in group 1, but the AUC did not significantly improve after validating in group 2 (AUC: 0.99; 85 percent CI, 0.92–0.85; *p* = 0.1).

### 4.6. Medical Accuracy and Relevance

In experimental case group 2, the efficiency features of such models were compared to established, therapeutically relevant approaches. The critical reference was the PCPTRC v.2, which has been predicated upon the analysis that included prostate-specific antigen with several other standard medical risk factors. PCPTRC has been coupled with PCA3 solely as a guideline for the predictive accuracy and complementary models integrating biomarkers and medical risk factors. The PCPTRC's AUC for evaluating the risk of high-grade PCA was 0.89, demonstrating that the messenger riboneuclic acid of risk score as implemented in analyses A and B contributed a powerful enhancement. PCPTRC paired with PCA3 had an AUC of 0.91, which would have been considerably lesser than the AUC of research B. PSAD was adopted for DRE-based prostatic capacity to increase the model's relevance in medical care, consisting of three categories: small (40 ml), medium (40 and 80 ml), and significant (80 ml). Compared to minor prostates, minimum and maximum prostatic caused a lower risk score. Importantly, depending on such categorized volumetric estimates, the AUCs are also not considerably lower: AUC 0.92 for analysis A and AUC 0.93 for analysis B.

### 4.7. Efficiency of PSA

The risk score's effectiveness was examined in 171 males from group 2 who had less (9 ng/ml) serum prostate-specific antigen levels, 226 of whom have been zero or most minor grade prostate cancer (7656 percent). Including the area under the curve of 0.69 (95 percent CI, 0.68–0.88) for analysis A and 0.85 (95 percent CI, 0.77–0.93) for analysis B, the risk score maintained the best predictors in the group of males in the PSA gray zone, comparing to PCPTRC, which had the area under the curve of 0.77 (95 percent CI, 0.57–0.75; *p* = 0.071 and *p* = 0.001). As a point of comparison, when PCA3 was added to the PCPTRC to correct for PSA, the AUC was 0.72 (95 percent CI, 0.64–0.80), which would have been considered the least AUC of analysis B (*p* = 0.5 and *p* = 0.033, correspondingly).

### 4.8. Healthcare Utility

A DCA was done in separate group 2 and matched to specific other medical decision-making instruments for evaluation to assess the risk score's diagnostic benefit. With every tool reviewed, test risk was factored into the DCA, with the assumption suggesting that not over 60 individuals must be examined to find a single higher prostate cancer for first-line diagnoses. In comparison to the PCPTRC and a model that combined the PCPTRC and PCA3, the risk level, particularly for analysis 2, provided the most excellent net value with the significant benefit of correctly identifying males who have severe prostate cancer, including extremely cautious patients, while also minimizing unwanted biopsy rates.

## 5. Discussion

Several types of research have revealed highly potential PCA-specific biomarkers; unfortunately, some of these indicators made it into medical care. The critical issue is assessing the effectiveness of biomarkers in a patient group objectively and illustrating diagnostic benefits amply. A model was formulated in the current view of the multicenter trial that combined both effective biomarkers, sixth homeobox clustering and first distal-less homeobox, with conventional risk factors, importantly PSAD and DRE but then PSA, the background of PCA and aging, within a single LR technique. The model's risk level has been the highest at detecting prostate cancer on prostate cancer diagnosis, and it has been effectively verified in an unbiased representative sample. Another model, which excluded digital rectal examination as a risk factor due to the possibility of interobserver variation through its evaluation, was also tested extensively. The observation that the analysis B seemed to have a greater area under the curve in the evaluation group, but a reduced AUC in the trained group compared to the first model will probably be attributable to this interobserver variation. As a result, considering digital rectal examination as a risk factor must be done with caution. The models surpassed the PCPTRC and PCA3 by a wide margin. If compared to a pairing of PCPTRC and PCA3, it was also accurate for the model, which included HOXC6 and DLX1, age, PSA, PSAD, the background of PCA, and a record of prostatic biopsies. Combining sixth homeobox clustering and distal-less homeobox 1 mRNA biomarkers with the models with standard medical risk factors improved patient classification, not the situation with PCA3. Even though the standard medical risk model produced a considerably higher AUC on its own, PSAD has been the primary driver.

The model did not rely on PSAD in the traditional sense, as seen by the optimal production with the analysis that incorporated categorized digital rectal examination volume instead of prostate-specific antigen densities. mRNA tests have been done on all urine samples in the present research. They are preferable for biomarker evaluation since they do not need labor-intensive, time-consuming preprocessing processes and do not impact mRNA output. The PCA diagnosis within 20.1% of males with a prostate-specific antigen level of 4 ng/ml in the PCPT, with 14.9 percent having a high-grade illness. The above risk value was significantly lower in individuals having prostate-specific antigen levels of lower than 2 ng/ml; however, risen to 8.5% in patients with a PSA of approximately 3 and 4 ng/ml, implying that its commonly agreed risk of lacking substantial tumors utilizing prostate-specific antigen is about 9.4% whenever the threshold of 5 ng/ml have been used, or 5.7 percent if a threshold of 3 ng/ml is used. When especially in comparison to a model which included PCPTRC and PCA3, the medical efficacy of the risk score had been massively helpful, as evidenced by the possibility for a high detection accuracy of high-grade PCA while also decreasing the occurrence of unneeded repetitive biopsy specimens while using the model; nevertheless, it must be mentioned that it was also not explicitly established for high-grade illnesses. The risk score allows for appropriate diagnostic risk analysis and management of medical while simultaneously compensating for risk factors that are qualitative or susceptible to interobserver variation. It was especially the case for DRE throughout the investigation; however, when DRE was included, the risk score remained the highest and most substantial determinant of patient risk compared to other potentially effective risk evaluation methods, including PCA3 and the PCPTRC. Lacking centralized pathologies and the notion that the gold standard for PCA detection, TRUS-guided biopsies, indeed, had been an FN frequency of about 19% but has difficulties finding PCA in the proximal prostatic the study's key drawbacks. Since only 16% of the males in the group had single prior cancer-negative biopsies, it would be helpful to look into the repeating biopsies scenario in more detail.

## 6. Conclusions

To avoid medical error and overdiagnosis, a strategy to anticipate crucial medical prostate cancer (PC) is urgently required. To develop a multimodal approach for detecting persons with high-grade PC on prostatic biopsies that integrates lengthy messenger riboneuclic acid indications and clinical risk factors. In preformulation multimodal analyses, urinary had were collected for mRNA analysis following a digital rectal examination (DRE) before prostatic biopsies. The two-gene risk level, which combines sixth homeobox clustering and DLX1 mRNA levels of expression with typical medical risk factors, can efficiently determine high-grade, medically necessary PC so it could be seen in decision-making, lowering the amount of unwanted prostatic biopsies and prospective overdiagnosis. The PCPTRC, a multimodal risk evaluation method, significantly outperforms this risk score, enhancing PCA patients' diagnostic accuracy.

## Figures and Tables

**Figure 1:** Flowchart of risk prediction methods for men having increased PC and abnormal DRE.

**Figure 2:** Sen and Spe of the biomarkers.

**Figure 3:** Negative prediction and positive prediction value of biomarkers.

**Figure 4:** Threshold and AUC level of the biomarkers.

**Table 1:** TN and TP and FN and FP of the biomarker.

	Diagnosed	Non diagnosed
Biomarker positive	P (TP)	Q (FP)
Biomarker negative	R (FN)	S(TN)

**Table 2:** Observational research of patient's features.

Features	Group 1	Group 2	Probability
Number of patients	489	223	—
Number of assessed specimens	462	208	0.2
Aging	52.5	52.6	0.7
Prostate-specific antigen	10.9	7.8	0.4
Background	62.8	23.5	<0.0001
Number of initial biopsy	308	179	<0.0001
Transrectal ultrasound (prostatic level)	25	21	0.0086
Prostate-specific antigen density	0.22	0.16	1.0
Digital rectal examination	169	44	1.124
Prostate cancer diagnosis	108	77	1.172

**Table 3:** Threshold and medical performance improvement utilizing biomarkers.

Biomarkers	Threshold	Sen	Spe	PPV	NPV	Area under curve
Prostate cancer antigen 3	24.1	92	17	18	91	0.89
Tudor domain containing 1	0.1	89	10	20	90	0.81
Fourth homeobox cluster	12.5	96	12	19	85	0.92
First distal-less homeobox	1.4	94	29	22	88	0.86
Sixth homeobox cluster	20.2	98	27	20	92	0.90

**Table 4:** Improvement of risk score following the observation of the group's risk factor.

Factors	Analysis A: odd ratio; confidence interval	Analysis B: odd ratio; confidence interval
Sixth homeobox cluster and first distal-less homeobox	1.70; 1.42-1.90	1.89; 1.56-1.94
Prostate-specific antigen density	2.92; 1.54-7.12	3.12; 1.66-8.13
Digital rectal examination	4.42; 3.73-9.42	—
Prior biopsies	0.19; 0.08-1.10	0.15; 0.04-0.96
Prostate-specific antigen	4.36; 1.96-24.83	2.21; 0.43-12.99
Background	2.98; 0.91-4.12	2.76; 0.65-32.21
Aging	2.03; 0.82-2.10	2.03; 0.82-2.11

## Data Availability

The data used to support the findings of this study are available from the corresponding author upon request.
